# Comprehensive Analysis of RAPGEF2 for Predicting Prognosis and Immunotherapy Response in Patients with Hepatocellular Carcinoma

**DOI:** 10.1155/2022/6560154

**Published:** 2022-04-26

**Authors:** Qing Wu, Yangzhi Hu, Qinghui Ma, Shanglin Yang, Junpeng Chen, Shunqian Wen, Guanqun Liao

**Affiliations:** ^1^Department of Hepatobiliary Surgery, Affiliated Foshan Hospital, Southern Medical University (The Second People's Hospital of Foshan), Foshan 528000, China; ^2^Department of Gastrointestinal Surgery, The Affiliated Hospital of Xiangnan University, Chenzhou 423000, China; ^3^Department of Oncology, Affiliated Foshan Hospital, Southern Medical University (The Second People's Hospital of Foshan), Foshan 528000, China

## Abstract

**Background:**

Hepatocellular carcinoma (HCC) is the sixth most common tumor worldwide. Additionally, deletion of RAPGEF2 plays a critical role in CNV and related to tumor immune microenvironment, whereas the prognostic potential of RAPGEF2 in HCC patient needs to be explored.

**Methods:**

We looked for prognostic potential genes in HCC using a variety of R programs. Then, using the LASSO Cox regression, we thoroughly evaluated and integrated the RAPGEF2-related genes from TCGA database. Meanwhile, utilizing TCGA and ICGA databases, the link between RAPGEF2 and immunotherapy response in HCC was studied. In vivo, the effect of RAPGEF2 on tumor development and the capacity of natural killer (NK) cells to recruit were confirmed. To ascertain the connection between RAPGEF2-related genes and the prognosis of HCC, a prognostic model was created and validated.

**Result:**

We demonstrated RAPGEF2 has a differential expression, and patients with deletion of RAPGEF2 gene get shorter survival in HCC. Additionally, the tissues without RAPGEF2 have a weaker ability to recruit the NK cells and response to immunotherapy. After that, we scoured the database for eight RAPGEF2-related genes linked with a better prognosis in HCC patients. Additionally, silencing RAPGEF2 accelerated tumor development in the HCC mouse model and decreased CD56+ NK cell recruitment in HCC tissues. TCGA database was used to classify patients into low- and high-risk categories based on the expression of related genes. Patients in the low-risk group had a significantly greater overall survival than those in the high-risk group (*P* < 0.001). Meanwhile, the low-risk group demonstrated connections with the NK cell and immunotherapy response. Finally, the prognostic nomogram showed a high sensitivity and specificity for predicting the survival of HCC patients at 1, 2, and 3 years.

**Conclusion:**

The prognostic model based on RAPGEF2 and RAPGEF2-related genes showed an excellent predictive performance in terms of prognosis and immunotherapy response in HCC, therefore establishing a unique prognostic model for clinical assessment of HCC patients.

## 1. Introduction

Hepatocellular carcinoma (HCC) is the sixth most commonly diagnosed cancer and the third leading cause of cancer death worldwide in 2020 [1]. Currently, the therapeutic options for HCC include surgical resection, transplantation, radiofrequency ablation, chemotherapy, and radiation [2]. In most cases, these treatments are ineffective for individuals with advanced hepatocellular carcinoma. According to a recent study, the inability to successfully treat HCC may be due to the disease's significant genetic variability [3]. Additionally, the molecular and clinical heterogeneity of HCC creates significant obstacles for tailored therapeutic therapy [4–6]. HCC patients may have variable prognoses and treatment responses based on their tumor cells' genetic heterogeneity, which has been extensively studied [7–9]. Therefore, finding the potential targets to predict the progress of HCC and treat the advanced HCC is needed.

Moreover, mounting data shows that copy number variants (CNVs) can significantly impact gene expression and are associated with illness risk. Studies have demonstrated that the expression of genes and cancer-related biological processes are affected by the presence or absence of CNVs [10]. Genomic structural variation known as CNV results in aberrant or normal variation in the number of copies of one or more portions of DNA, depending on the gene [11]. Previous study showed the deletion of GATA4 gene was the most prominent feature in all HCC [12]. Additionally, Hippo, Wnt/*β*-catenin, and Notch pathways form an interacting network to suppress tumorigenesis in HCC [13]. Although Rap2, a member of Ras GTPase family, can regulate the Wnt/*β*-catenin pathway and Hippo pathway, respectively [14, 15], the mechanism underlying its function of Rap2 in HCC remains poorly understood. As the Rap2 activator [15–17], Rap guanine nucleotide exchange factor 2 (RAPGEF2) can activate Rap2 resulting in inhibition of YAP and TAZ to control the mechanosensitive cellular activities [15]. However, the prognostic value of RAPGEF2 and the relationship between RAPGEF2 and tumor immune microenvironment remain unknown.

In this study, RAPGEF2 has been shown to be an important prognostic biomarker for HCC patients by screening data from both TCGA and ICGCC databases. Our findings indicate that RAPGEF2 and RAPGEF2-related genes are more predictive of prognosis and immunotherapy response in HCC than other genes.

## 2. Method and Material

### 2.1. The Copy Numbers Were Acquired from TCGA Database

A total of 374 HCC samples and 50 normal tissue samples were obtained from TCGA (https://portal.gdc.cancer) and ICGC databases, respectively, for RNA sequencing and analysis (https://dcc.icgc.org/, including 231 HCC samples). The copy number variation data of HCC patients was also downloaded from TCGA cohort. Research conducted in the current study adhered to TCGA and ICGC database access rules and publishing requirements.

### 2.2. Survival Analysis and Construction of Prognostic Model

The Kaplan-Meier curve was plotted by the “survminer” R package between different groups in TCGA cohort. And the “limma” R package was used to identify the differentially expressed levels between different groups. Coexpression analysis was also conducted to identify correlation genes through limma package. To identify genes with prognostic value, a univariate Cox analysis of overall survival (OS) was done using the R package “survival.”

The “glmnet” R program was used to include the prognostic genes into the LASSO Cox regression. To avoid the model overfitting, the penalty regularization parameter *λ* was set using tenfold cross-validation. Each patient was assigned a risk score based on the following formula: risk score = ∑_*i*=1_^*n*^(Expi∗*βi*). In this example, we have *n* genes, Expi is the expression value of gene *i*, and *βi* is the coefficient of gene *i* derived using LASSO regression analysis. Univariate and multivariate Cox regression analyses were used to examine if the risk score was an independent predictive predictor of OS when compared to other clinical characteristics.

The R package “rms” was used to create a predictive nomogram and associated calibration maps based on independent predictive criteria. The “timeROC” R program was used to run a receiver operating characteristic (ROC) curve analysis to determine the prognostic model's accuracy in predicting future events.

### 2.3. Functional Enrichment Analysis and Immunotherapy Response Predictions

Using single-sample gene set enrichment analysis (ssGSEA) and the “gsva” R package, researchers assessed the infiltration score of 16 immune cells and the activity of 13 immune-related pathways.

With tumor immune dysfunction and exclusion (TIDE) (http://tide.dfci.harvard.edu/), an expression signature of T cell malfunction and exclusion is integrated into a computational model of tumor immune evasion. The TIDE algorithm was used to predict the clinical response of HCC patients to immune checkpoint blockade (ICB).

### 2.4. Cell Culture and Transfection

The American Type Culture Collection (ATCC) provided MHCC97 cells growing in RPMI-1640 medium with 10% fetal bovine serum (FBS; ExCell Bio, Shanghai, China). Mycoplasma contamination was found in these cell lines. The manufacturer's instructions were followed while transfecting cells using Exfect 2000 transfection reagent (Vazyme, NJ, China).

### 2.5. Lentivirus and Stable Cell Line Generation

MHCC97 cells were cotransfected with mouse RAPGEF2 shRNA (cat. KN422055, Origene) plasmid, psPAX2, and pCMV-VSV-G, and the supernatant containing lentivirus particles was collected at 48 hours after transfection, when the cells had been infected with these three things. To generate a cell line stably expressing RAPGEF2 shRNA, MHCC97 cells were expanded to 50-80% confluence prior to lentiviral infection and then treated with 1-3 *μ*g/ml puromycin 24 h later. Western blot analysis was used to select stable clones and to determine the expression of RAPGEF2.

### 2.6. Western Blot

Cells were lysed with RIPA buffer supplemented with protease inhibitors and phosphatase inhibitors for 30 min on ice. Cell lysates were centrifuged for 15 min at 1.2 × 10^4^ rpm, 4°C. The Pierce BCA protein assay kit was used to measure the total protein concentrations. Equivalent quantities of protein were isolated and transferred to PVDF membranes using 10% SDS polyacrylamide gels [18]. The membranes were blocked with 5% BSA dissolved in TBST for 1 h and then incubated with primary antibodies (RAPGEF2, cat. NBP2-88124, Novus) for overnight at 4°C. After washing, the membranes were incubated with peroxidase-conjugated secondary antibodies for 1 h at room temperature. Immune-reactive bands were visualized by Clarity^TM^ Western ECL Substrate. Gray values for each band were measured using the Image J software.

### 2.7. HCC Xenograft

Hangzhou Ziyuan Experimental Animal Technology Co., Ltd (Hangzhou, China) offered four- to six-week-old BALb/c nu/nu male mice. All studies were conducted in accordance with the guidelines established by the Guangdong Medical Animal Experiment Center. The mice were maintained in an infection-free environment. Without using any selection criterion, mice were randomly separated into independent groups of ten (*n* = 10). All BALb/c nu/nu mice were subcutaneously infected with 2 × 10^6^ MHCC97 cells that expressed control (Ctrl) and RAPGEF2 shRNA. Tumor development was tracked, and tumor volumes were determined using the formula *V* = (*LW*^2^)/2 (*L*: length and *W*: width) as published before. The investigator was not blinded throughout the experiment or while evaluating the results.

### 2.8. Flow Cytometry

Cells were collected, resuspended in a flow cytometry staining buffer, and distributed into 1.5 mL EP tubes. Following fixed with 4% paraformaldehyde on ice and permeabilized with 0.1% Triton X-100 in PBS for 5 min, the cells were incubated with indicated Alex Fluor-conjugated antibodies (CD3, Novus, NBP2-25186 and CD56, Novus, NBP2-15186) for 1 h on ice and analyzed by FlowJo (BD Biosciences, San Jose, CA).

### 2.9. Statistical Analysis

All statistical analyses were conducted using the R programming language (Version 4.0.3). A Kaplan-Meier analysis and a log-rank test were used to compare the OS of various groups. All *P* values were calculated with a two-tailed distribution. If not otherwise mentioned, a *P* value of 0.05 was deemed statistically significant.

## 3. Result

### 3.1. Estimation of Expression of RAPGEF2 in the HCC

Screening from TCGA database, we can get the Kaplan-Meier curve that the patients with high RAPGEF2 expression had longer survival than the low RAPGEF2 expression in HCC (*P* = 0.001) (Figure 1(a)). We initially analyzed the frequency of copy number variations (CNVs) and somatic mutations of RAPGEF2 gene in HCC patients. There were about 42.4% of patients that had the deletion of CNV alteration of RAPGEF2 gene on chromosomes, while the increase was less than 4% (Figure 1(b)). Meanwhile, the patients with RAPGEF2 deletion had longer OS than the normal (Figure 1(c)). To confirm the influence between the expression of the RAPGEF2 gene and the deletion, we analyzed TCGA database for different expression. The results showed that the deletion of RAPGEF2 influenced straightly the expression of the RAPGEF2 gene (Figure 1(d)).

### 3.2. Estimation of the Role of RAPGEF2 in Tumor Immune Microenvironment and Cancer Immunotherapy Response in HCC

To evaluate the relationship between tumor immune microenvironment and the deletion of RAPGEF2, we analyze the different evaluation indicators, like the recruitment of immune cell, TMB, TIDE, and the response for the immunotherapy. The result revealed that the group of RAPGEF2 deletion has weaker ability to recruit the natural killer (NK) cell and tumor-infiltrating lymphocytes (TILs) than the normal group (Figure 2(a)). And the TMB in the RAPGEF2 group is less than the normal (Figure 2(b)). For the estimation of immunotherapy, we also found in the group of RAPGEF2 deletion, the TIDE value was higher, and the ability of immune response was decreased (Figures 2(c) and 2(d)).

### 3.3. RAPGEF2 Knockdown Promoted Tumor Growth and Supressed the Infiltration of CD56+ NK Cells

To further discover the potential influence of RAPGEF2 on HCC progression in vivo, we established human MHCC97 HCC cell stably expressing control (Ctrl) or RAPGEF2 shRNA where the RAPGEF2 protein was successfully knocked down (Figure 3(a)) and implanted MHCC97 cells with or without RAPGEF2 knockdown into BALB/C nu/nu mice. To investigate the effect of RAPGEF2 on tumor growth, we noticed that silencing RAPGEF2 enhanced tumor growth (Figure 3(b)) and raised tumor weight (Figure 3(c)) much more than cells expressing Ctrl shRNA. To verify the relationship between RAPGEF2 and CD56+ NK cells in HCC, we found knockdown RAPGEF2 in HCC cells reduces tumor infiltrating CD56+ NK cell recruitment in MHCC97 xenograft tumors (Figures 3(d) and 3(e)).

### 3.4. Constructing and Validating a Risk Model for HCC Based on RAPGEF2-Related Genes

To find the underlying mechanism, we screened RAPGEF2-associated prognostic genes (correlation coefficient > 0.5) in TCGA using univariate Cox regression analysis. Sixteen RAPGEF2-related genes in TCGA dataset were significantly correlated with OS (Figure 4(a)). Then, we enhanced the forecast accuracy and explainability of the statistical model by the LASSO-penalized Cox analysis and established the risk scoring system analyzing expression profile. This technique efficiently identifies the most relevant prediction signals and generates a prognostic indicator that may be used to anticipate clinical outcomes. The dashed perpendicular line depicts the log first-rank value of log *λ* with the least segment probability bias. Hence, RAPGEF2 and RAPGEF2-related genes were selected for the subsequent multivariate analysis (Figures 4(b) and 4(c)). The risk score was calculated as follows: risk score = SUM (SMARCAD1∗0.596 − SORBS2∗0.118 + ZNF148∗0.493 − RAPGEF2∗0.512 − AKAP13∗0.539 − PIK3R1∗0.0939 + ARID1A∗0.397 − CTSO∗0.00274 − GNE∗0.140). The Kaplan-Meier curve demonstrated that low-risk patients had a better prognosis than high-risk patients (Figure 4(d), *P* < 0.001), indicating that the prognostic signature had a high sensitivity and specificity for predicting OS. Additionally, a significant correlation was identified between the nine genes and the prognosis of HCC patients. Additionally, the ROC analysis revealed that RAPGEF2 and RAPGEF2-related genes had a significant predictive value for patients with HCC in TCGA dataset. (1-year AUC = 0.771, 2-year AUC = 0.731, and 3-year AUC = 0.744; Figure 4(e)). To verify the reliability of the risk score model, we analyzed another group of patients from the ICGA database (Figure 4(f)). The results from TCGA were comparable, indicating that these genes have a strong and consistent ability to predict OS.

### 3.5. Immune Infiltration and Immunotherapy Responses in Individuals with Varying Degrees of Risk

To examine the relationship between risk score, immunological state, and immunotherapy, we measured risk scores for various immune cell subsets, cell functions, linked pathways, and immunotherapy. The results indicated that high-risk patients' NK cell counts were lower than those in the low-risk group (Figure 5(a)). In TCGA database, there were substantial variations between the two groups in type I and type II interferon response (Figure 5(b)). In the ICB response, we found the high-risk patients have the higher TIDE value than the low-risk in TCGA database (Figure 5(c)), which predicted the outcome of cancer patients treated with immunotherapy more accurately than other biomarkers [19]. Therefore, we observed the response for immunotherapy and found the high-risk patients get worse immunotherapy response (Figure 5(d)). Both results in these two aspects were verified in the ICGA database (Figures 5(e) and 5(f)).

### 3.6. Construction and Validation of the Predictive Nomogram

We examined the model using univariate and multivariate Cox regression analyses of other clinical variables (including gender, age, and TNM stage) to see if it was independent of other clinical prognostic factors that may impact the patients' prognosis. TNM stage (HR = 1.433) was found to be an independent predictor of OS (Figures 6(a) and 6(b)). Individual survivability for 1, 2, and 3 years might be quantified using a nomogram constructed from these independent prognostic biomarkers. The nomogram's C-index was 0.719 (95% CI: 0.668–0.769). The calibration curves revealed a high degree of congruence between expected and observed OS at 1, 2, and 3 years (Figures 6(c) and 6(d)). Meanwhile, the nomogram's predictive value was validated using ROC curves. In TCGA database, the AUCs for 1-, 2-, and 3-year OS were 0.785, 0.748, and 0.774, respectively (Figure 6(e)), as the similar results tested in the ICGA database (AUC: 1-, 2-, and 3-year OS were 0.769, 0.715, and 0.698) (Figure 6(f)).

## 4. Discussion

In this study, we analyzed the expression of RAPGEF2 gene and eight RAPGEF2-associated genes (SORBS2, SMARCAD1, ZNF148, AKAP13, PIK3R1, ARID1A, CTSO, and GNE) in HCC sample and investigated their relationship with OS of HCC patients and the immunotherapy response using TCGA and ICGC databases. Patients with the deletion of RAPGEF2 had shorter OS, higher TIDE value, and worse immune response. Finally, we developed a prognostic nomogram based on these genes that demonstrated high sensitivity and specificity for predicting OS and its connection with immunotherapy response. Our work showed that these RAPGEF2-related genes can be used as predictive biomarkers in HCC. Meanwhile, it is the first predictive model based on RAPGEF2 and RAPGEF2-associated genes for HCC patients.

Currently, using Genomic Identification of Significant Targets in HCC, it was discovered that focused CNVs may be further identified. The findings discovered recurrent HBV integration events at the known and potential cancer-related TERT, MLL4, and CCNE1 genes, which demonstrated increased gene expression in HCC compared to normal tissue [20]. Our study also proved the deletion of RAPGEF2 was associated with HCC patients' survival. Meanwhile, we initially analyzed the relationship between RAPGEF2 and tumor immune microenvironment. The ability concerning both recruitment of NK cells and TIL and the response for the immunotherapy get weaker in HCC tissues with RAPGEF2 deletion. NK cells have been demonstrated to be cytotoxic to tumor cells in a variety of malignancies, including HCC [21–23]. Increased NK cell density in malignancies correlates with tumor response to anti-PD1 treatment [24, 25]. Previous studies found HCC-derived exosomes, circUHRF1, inhibited NK cells function by upregulating the expression of T cell immunoglobulin and mucin domain 3 (TIM-3) via degradation of miR-449c-5p, which may drive resistance to anti-PD1 immunotherapy in HCC patients [26]. And targeting circUHRF1 might recover the sensitivity of HCC to anti-PD1 therapy [26]. As further research shows, hypoxic stress in HCC tissues, activation/inhibition of NK receptor (NKR) switches, and the effect of immunomodulatory components in TME are all major contributors to NK cell dysfunction, which is strongly linked to antitumor immune exhaustion and poor prognosis [27, 28]. Several early clinical studies indicated that postoperative HCC patients with a high amount of lymphocyte infiltration, particularly T cells, had a lower rate of recurrence and a better prognosis [29]. Our result demonstrated the similar result that the RAPGEF2 deletion patients get less NK cells, TIL, and worse survival and immunotherapy response. However, the underlying regulatory role among them remains further investigated.

Additionally, we also built a prognostic nomogram to analyze the RAPGEF2-associated genes, and the result was the same as the single gene. The patients with low score had the longer survival, better recruitment of NK cells, and better response for the immunotherapy. Previous studies found about 4–17% of HCCs had ARID1A alterations, and the ARID family may contribute to poor prognosis for the HCC [30–33]. In the ovarian clear cell carcinoma (OCCC), people discovered that ARID1A WT OCCCs enhanced Th1-type immune responses, cytotoxic T cell responses, and NK cell activation, but ARID1A mutant OCCCs lacked type II and type I IFN signaling pathways [34], but the latent mechanism needs to discover. The interferon family includes type I and type II interferons, which are implicated in antitumor and immune responses [35]. Our results also observed the same phenomena in type I and type II interferon responses, recruitment of NK cells, and response for the immunotherapy, which may be beneficial for the survival in HCC. Meanwhile, some studies showed the SMARCAD1 was involved in the different cancer, like the breast cancer [36] and pancreatic cancer [37]. We also found the expression of SMARCAD1 gets higher, the shorter OS in HCC. And the SORBS2 gene can suppress HCC metastasis through the c-Abl/ERK signaling pathway [38]. In our research, because the corresponding coefficient of SORBS2 is negative, the risk score would get less as the expression gets higher. Impaired gene influencing the immunity may be one of the reasons for poor prognosis in high-risk patients.

This is the first study that combines RAPGEF2 gene with clinical data to construct a prognostic model. However, several restrictions should be solved. To begin, we created and verified the prognostic model using publicly available data. Prospective real-world data are required to validate this model's therapeutic effectiveness. Additionally, the relationship between RAPGEF2-related genes and the immune microenvironment of tumors warrants additional exploration.

## 5. Conclusion

In summary, we proposed a novel prognostic model of RAPGEF2 and its associated genes in HCC, which had a critical prognostic value for immunotherapy response of HCC patients. Further researches need to focus on the mechanisms between these genes and tumor immune cells in HCC.

## Figures and Tables

**Figure 1:** Expression variation and survival curves of RAPGEF2 genes in hepatocellular carcinoma (HCC). (a) Kaplan-Meier curves for the OS of patients in the different RAPGEF2 expression from TCGA database. (b) The location of copy number variation (CNV) alteration of RAPGEF2 on chromosomes using TCGA datasets. (c) The Kaplan-Meier curves for the OS of patients between the deletion and normal of RAPGEF2 expression from TCGA database. (d) The expression of RAPGEF2 in different tissues.

**Figure 2:** Relationship among RAPGEF2, immune infiltration tumor immune dysfunction exclusion, and immunotherapy response to HCC patients. (a) The scores of 16 immune cells. (b) The scores of 13 immune-related functions. (c) The value of the tumor immune dysfunction and exclusion (TIDE). (d) The response to immunotherapy (^∗^*P* < 0.05; ^∗∗^*P* < 0.01; ^∗∗∗^*P* < 0.001; ns: no significant).

**Figure 3:** RAPGEF2 knockdown promotes tumor growth in HCC cancer xenografts. (a) Western blotting examination of MHCC97 cells transfected with either control (Ctrl) or RAPGEF2 shRNA. (b, c) The tumor growth curve and weights of the tumors were determined. (d, e) Fluorescence-activated cell sorting (FACS) study of CD56+CD3-natural killer cells in MHCC97 xenograft tumors with either control (Ctrl) or RAPGEF2 shRNA. Data represents the mean ± SD, *n* = 10 per group. ^∗^*P* < 0.05, ^∗∗^*P* < 0.01, and ^∗∗∗^*P* < 0.001.

**Figure 4:** Risk model and the Kaplan-Meier curves for the OS in HCC patients based on RAPGEF2 and its related genes. (a) The univariate Cox regression analysis demonstrated a substantial correlation between the identified genes and clinical prognosis. (b) To cross-validate the error curve, the tuning parameters (log *λ*) of OS-related proteins were selected. Perpendicular imaginary lines were drawn at the ideal value using the minimum and 1-se criterion. (c) The LASSO coefficient profile of 13 OS-associated genes was drawn together with the perpendicular imaginary line at the value determined by 9-fold cross-validation. (d) Kaplan-Meier curves for the OS of patients in TCGA database who were classified as high-risk or low-risk. (e) ROC analysis using TCGA database. (f) ROC analysis using the ICGC database.

**Figure 5:** Relationship among risk model, immune infiltration tumor immune dysfunction exclusion, and immunotherapy response to HCC patients. (a) The scores of 16 immune cells. (b) The scores of 13 immune-related functions. (c) The value of the TIDE from TCGA database. (d) The response to immunotherapy from TCGA database. (e) The value of the TIDE from ICGC database. (f) The response to immunotherapy from ICGC database. (^∗^*P* < 0.05; ^∗∗^*P* < 0.01; ^∗∗∗^*P* < 0.001; ns: no significant).

**Figure 6:** Predictive nomogram construction and validation. (a) The univariate Cox regression analysis's results. (b) The multivariate Cox regression analysis's results. (c) A nomogram for predicting the 1-, 2-, and 3-year OS of patients with HCC. (d) Nomogram calibration curves for OS prediction at 1, 2, and 3 years. (e) ROC analysis using TCGA database. (f) ROC analysis using the ICGC database.

## Data Availability

The corresponding author may provide the data and materials used to support the conclusions of this study upon request.
